# Effects of Etanercept on TNF-*α* Inhibition in Rats with Adenine-Induced Chronic Kidney Disease

**DOI:** 10.1155/2022/4970753

**Published:** 2022-05-19

**Authors:** Edgar Mendieta-Condado, Elda Cristina Villaseñor-Tapia, Francisco Javier Gálvez-Gastelum, Irinea Yáñez-Sánchez, Oscar Pizano-Martínez, Alejandro Canales-Aguirre, Ana Laura Márquez-Aguirre

**Affiliations:** ^1^Departamento de Control de Calidad, Laboratorio Estatal de Salud Pública, Secretaría de Salud Jalisco, 46170 Zapopan, Jalisco, Mexico; ^2^Unidad de Biotecnología Médica Farmacéutica, Centro de Investigación y Asistencia en Tecnología y Diseño del Estado de Jalisco, Mexico; ^3^Laboratorio de Patología, Departamento de Microbiología y Patología, Centro Universitario de Ciencias de la Salud, Universidad de Guadalajara, Mexico; ^4^Centro de Investigación en Nanociencias y Nanotecnología, Departamento de Ciencias Naturales y Exactas, Centro Universitario de los Valles, Universidad de Guadalajara, Mexico; ^5^Instituto de Investigación en Reumatología y Sistema Músculo Esquelético, Departamento de Morfología, Centro Universitario de Ciencias de la Salud, Universidad de Guadalajara, Mexico

## Abstract

**Introduction:**

Chronic kidney disease (CKD) constitutes a chronic inflammatory state associated with an increase in inflammatory mediators and profibrotic molecules such as tumor necrosis factor-*α* (TNF-*α*). Etanercept (ETA) is a TNF inhibitor widely used in treatment of autoimmune inflammatory diseases. However, the effects of TNF-*α* inhibition in the establishment of CKD have not been fully elucidated. We evaluate the effects of TNF inhibition by ETA in adenine- (Ad-) induced CKD in rats.

**Methods:**

Rats were divided into three groups: control, renal injury model, and model plus ETA (2 mg/kg, 3 times per week (w); sc). Renal injury was induced by Ad administration (100 mg/kg, daily for 2 or 4 w; orogastric). Serum TNF-*α* levels and biochemical parameters for renal function were evaluated. Histopathological changes in the kidney were assessed using H&E and Masson's trichrome staining and also immunostaining for tubular cells.

**Results:**

Ad administration produced a renal functional decline, tubular atrophy, interstitial inflammation, and fibrosis for 2 w, followed by renal anemia, several renal dysfunctions, tubular atrophy, and fibrosis at 4 w. A significant increase in serum TNF-*α* levels was observed from 2 w of Ad administration and remained elevated up to 4 w. Treatment with ETA partially reduced kidney damage but was very effective to blocking serum TNF-*α*.

**Conclusion:**

Although inhibition of TNF by ETA was very effective in reducing serum TNF-*α*, this strategy was partially effective in preventing Ad-induced CKD.

## 1. Introduction

Chronic kidney disease (CKD) is characterized by irreversible tissue damage, decrease of renal function, and progressive histological changes in the kidney [1]. CKD constitutes a chronic inflammatory state with the elevation of several inflammatory mediators such as IL-1*β*, IL-1RA, IL-6, tumor necrosis factor alpha (TNF-*α*), and C-reactive protein (CRP) [2]. Inflammation plays a critical role in the initiation and progression of renal fibrosis [3].

TNF-*α* is an inflammatory cytokine produced mainly by immune cells such as macrophages/monocytes, and its biological activity depends on binding to its receptors [4]. There are two distinct receptors for TNF (TNFRs): a 55-kilodalton protein (p55) and a 75-kilodalton protein (p75), and the role of both TNF-*α* and TNFRs in renal dysfunction has been described previously [5, 6].

TNF inhibitors (TNFi) are used clinically to counterbalance the high TNF levels in several autoimmune rheumatic diseases such as rheumatoid arthritis (RA) [7, 8]. Interestingly, treatment of RA with TNFi has been associated with lower risk on incident CKD [9, 10].

Etanercept (ETA) is one of the registered TNFi (DrugBank accession DB00005). It is a fusion protein that is composed of the extracellular ligand-binding portion of human p75 TNFR linked to the Fc portion of human IgG1 and acts as a “TNF decoy receptor” by inhibiting the binding of soluble TNF-*α* to its cell surface receptor [11]. Some studies have reported the effectiveness of ETA-reducing inflammation in different pathologies related with an exacerbated immune response or fibrosis [12–14]. However, the impact of TNF-*α* inhibition on CKD progression is not fully elucidated.

The chronic adenine (Ad) diet model results in renal dysfunction. Ad is metabolized to 2,8-dihydroxy-adenine which forms crystalline casts within the renal tubules. This induces progressive kidney damage characterized by tubular atrophy accompanied by chronic interstitial inflammation and fibrosis [15–17].

In this study, we employed the adenine-induced chronic kidney disease (Ad-CKD) model to produce rapid-onset kidney disease in rats to assess the effects of ETA on TNF inhibition and its impact on progressive kidney failure.

## 2. Materials and Methods

### 2.1. Animals and Treatment

Thirty male Wistar rats weighing approximately 200 g were purchased from Bioterio Morelos. Rats were maintained under SPF conditions with a room temperature of 22–26°C and humidity of 50–60% under a 12 h light/dark cycle, with access to standard food and water *ad libitum*. Animal procedures were approved by the Institutional Animal Care and Use Committee (CIATEJ protocol number 2019-009A).

Rats were randomly divided into three groups (*n* = 10 per group): control, kidney damage (Ad), and kidney damage plus etanercept (Ad+ETA). The control group received orogastric administration of water and a subcutaneous (sc) injection of normal saline, both vehicles of Ad and ETA, respectively. Kidney damage was carried out by orogastric administration of Ad (Sigma, A8626) at a dose of 100 mg/kg daily for 4 weeks, with a cutoff preliminary at 2 weeks [15, 16]. Etanercept (Enbrel® 50 mg) was administrated by sc injection at a dose of 2 mg/kg, 3 times per week one hour before the dose of Ad. This dose was selected as an average of previous studies reporting antifibrotic effects of ETA [12–14].

### 2.2. Analysis of Hematological and Biochemical Parameters

Hematic biometry encompasses erythrocyte count, hemoglobin, and hematocrit levels determined by the impedance method. Biochemical tests were carried out to count the levels of serum creatinine (sCr), urine creatinine (UCr), serum urea (sUr), and blood uremic nitrogen (BUN) by means of dry chemistry, in order to evaluate the renal function. Glomerular filtration rate (GFR) was determined using the levels of sCr, UCr, urinary flow, and average kidney weight, using the formula: ((uVol (ml/min) × UCr)/sCr)/average kidney weight (g) [18].

### 2.3. Histopathological Analysis

Kidney samples were fixed in 4% paraformaldehyde; one part was dehydrated and embedded in paraffin. Tissues were sectioned (5 *μ*m) with a microtome and then stained with hematoxylin and eosin (H&E) or Masson's trichrome following standard protocols. Determination of inflammatory infiltrate, tubular damage, and fibrosis was performed by a double-blind semiquantitative analysis. We observed 23 slides, with 2 tissues in each one and 15 fields at 10x and 40x approach for each one. Then, we assessed a score of percentage of damage, inflammation, and fibrosis. The scale considered 0-4 scores or levels according to percentage, where 0 represents the absence or no damage, 1 represents the little presence or minor damage (<25%), 2 represents the presence or damage in approximately the middle of the field (25-50%), 3 represents the presence or damage in approximately two-thirds of field (50-75%), and 4 represents the presence or damage in the entire field (>75%) [19, 20].

Another section of the fixed kidneys was cryoprotected (30% sucrose in PBS, pH7.4) overnight at 4°C and then was embedded in Tissue-Tek (O.C.T. Compound Sakura) and snap frozen at -25°C. Frozen tissues were sectioned (10 *μ*m) with a cryostat for immunofluorescence. Tissues were stained with antibody for Thy-1 (CDw90) (Santa Cruz Biotechnology, sc-6071) at a dilution of 1 : 250 overnight at 4°C, washed, and then incubated with a secondary antibody, Alexa Fluor® 488 (Invitrogen, A32814). Nuclei were counterstained with DAPI (Invitrogen, 62248). Images were obtained with confocal microscopy (Leica TCS SPE DM5500, software LAS X) at a 40x magnification; 3 cortical fields were analyzed per sample.

### 2.4. Determination of TNF-*α* Concentration in Serum

Serum levels of TNF-*α* were quantified by a commercial ELISA kit, according to the supplier's instructions (Sigma, RAB0479). Results were analyzed by linear regression adjustment, using the standard concentrations of TNF-*α* and the absorbance given at 450 nm.

### 2.5. Statistical Analysis

Statistical analysis was performed using GraphPad Prism version 5 (San Diego, CA, USA). One-way ANOVA was used followed by Dunn's multiple comparison posttest. The statistically significant differences of the results with a *P* value ≤ 0.05 were considered. Results are represented as the mean ± standard error (SEM).

## 3. Results

### 3.1. Treatment with ETA Reduces Serum Levels of TNF-*α* in Rats with Kidney Damage

To demonstrate the TNF inhibition by ETA, we performed an ELISA assay to quantify the levels of TNF-*α* in serum. Ad administration significantly increased serum TNF-*α* levels from the second week (570 pg/ml), and they remained high until the fourth week of Ad administration (587 pg/ml) compared to the control (104 pg/ml). Treatment with ETA (Ad+ETA) significantly decreased TNF-*α* concentrations from week 2 (137 pg/ml) to week 4 (125 pg/ml), compared to the Ad groups without treatment shown in Figure 1.

### 3.2. Partial Recovery of Kidney Function in Rats with ETA Treatment

First, the kidney appearance was observed. As shown in Figure 2(a), the kidney of the Ad groups differed markedly for the control. Macroscopic changes in the kidney were observed since the second week and persist until fourth week. The kidneys were grossly enlarged, and color change was yellowish with small surface nodules. It is important to note that this enlargement of the kidneys occurred despite the fact that all the animals with Ad administration significantly decreased their weight gain versus the control, although the Ad+ETA group gained more weight compared to the untreated Ad group at both 2 and 4 weeks (Figure 2(b)). In the model group, Ad-CKD (Ad 4 w) kidney is reaching a significant enlargement with a weight of 4.2 g and a length of 2.9 cm versus the control (1.1 g and 1.7 cm). A recovery in weight and size was observed in the Ad+ETA group at fourth week (3.3 g and 2.4 cm, respectively) versus the Ad group (Figures 2(c) and 2(d)).

Next, hematological and biochemical analyses were performed to evaluate renal anemia and kidney function. Chronic kidney damage depletes the number of EPO-producing cells in the kidney; therefore, hemoglobin, hematocrit, and erythrocyte indexes descend. Ad significantly decreased hematic parameters at 4 weeks; however, treatment with ETA did not have an impact on these (Table 1). Moreover, serum creatinine (2.9 ± 0.34 mg/dl), serum urea (276.3 ± 25.1 mg/dl), blood urea nitrogen (BUN) (129.2 ± 11.7 mg/dl) levels, and urinary volume 24 h (41.3 ± 4.7 ml) were significantly increased in animals with Ad, compared to the control group (0.32 ± 0.02 mg/dl, 33.8 ± 1.6 mg/dl, 15.9 ± 0.75 mg/dl, and 11 ± 5.7 ml, respectively) (Figures 3(a), 3(b), 3(c), and 3(e)), while urinary creatinine (68.1 mg/dl) and GFR (0.02 ml/min/g kidney) were significantly decreased in animals with Ad, compared to the control group (119.1 ± 11.3 mg/dl, 0.266 ± 0.03 ml/min/g kidney) (Figure 3(d), Table 1). Interestingly, some of these parameters were improved with ETA treatment. Serum creatinine (2.2 ± 0.26 mg/dl), serum urea (209.6 ± 25.9 mg/dl), and BUN (97.9 ± 12.1 mg/dl) levels were significantly decreased in the Ad+ETA group compared to the Ad group at 4 weeks (Figures 3(a), 3(b), and 3(c)), although there were no differences between the Ad and Ad+ETA groups in urinary creatinine, urinary volume, or GFR (Figures 3(d) and 3(e), Table 1).

Treatment with ETA partially reduces kidney damage prior to the establishment of CKD. Adenine administration produces a persistent inflammation and a progressive scarring evolution to CKD. We found a large accumulation of inflammatory infiltrate in kidney tissue from the second week with a score 3 (62%) and reaching to score 4 (79%) at the fourth week in groups with Ad. The administration of ETA partially decreased the percentage of inflammatory infiltrate by approximately 10% at second week (54%) but only in 3% at 4 weeks (76%), shown in Figure 4(a). Similarly, it was observed that the administration of Ad generated alterations in the renal tubular structure, such as tubular atrophy with interstice expansion and loss and flattening of tubular epithelial cells in the second week with a score 2 (50%) and reaching to score 3 (74%) at four weeks. Treatment with ETA decreased tubular damage by 10% at week 2 with a score 2 (40%) and 17% at week 4 with score 3 (57%) compared to the group without treatment, shown in Figure 3(a). Additionally, in the immunostaining for tubules, we observed a loss of Thy-1 labeling in the groups with Ad compared to the control from two weeks, this loss of labeling being more evident at four weeks, although it seems that treatment with ETA maintains the expression of Thy-1 in the proximal tubules at four weeks (Figure 4(b)). Moreover, the administration of Ad caused peritubular fibrosis from the second week with score 3 (57%) and reaching to score 4 (80%) at the fourth week. Treatment with ETA reduced the percentage of fibrosis by 18% in the second week (39%), but not at four weeks, when the CKD model is already established; both groups showed similar percentage of fibrosis (score 4, 80%) (Figure 4(c)).

## 4. Discussion

TNF-*α* is a potent proinflammatory cytokine and important mediator of inflammatory tissue damage. High serum levels of TNF-*α* are positively correlated with the severity of kidney injury [2]. In our study, the administration of Ad increased the serum levels of TNF-*α* concentration up to four times from week 2 and remained elevated until week 4, confirming the elevation of this cytokine in the Ad-CKD model. Similar data has been previously reported, where elevated levels of this cytokine were approximately 3 times more in the Ad group compared to the control [24]. Treatment with ETA significantly reduces circulating levels of TNF-*α* from the second week up to the fourth week. With these data, we demonstrated an efficient TNF-*α* inhibition by ETA. This finding is consistent with the action mechanism of ETA that inhibits binding of TNF to cell surface TNFRs, rendering biologically inactive TNF.

Moreover, in our study, we found a progressive deterioration of kidney function induced by Ad. According to previous studies [20, 21], renal anemia and reduced GFR occurred at 4 weeks after Ad administration. Interestingly, partial recovery of kidney function was observed in rats with ETA treatment. Serum creatinine, serum urea, and BUN levels were significantly decreased in the Ad+ETA group at 4 weeks.

In addition, as previously mentioned, it is well known that Ad administration induced renal toxicity associated with tubular injury and produced persistent inflammation and a progressive scarring evolution to CKD [16, 19, 22]. In accordance with this, in our study, we analyzed renal morphology and histology. A large amount of inflammatory infiltrate, tubular atrophy, and interstitial fibrosis was found from the second week of Ad administration and becoming severer at 4 weeks. An immunostaining to Thy-1 (CDw90) confirms the tubular atrophy in proximal tubular cells in the Ad groups and shows a protective role of ETA in kidney parenchyma cells. Overall, morphological observation and pathological staining showed that ETA ameliorated kidney injury in rats. ETA attenuated morphological changes and reduced inflammatory infiltrate, tubular atrophy, or interstitial fibrosis induced by Ad at 2 weeks. However, ETA treatment partially reduced inflammatory infiltrate or tubular atrophy, but was not effective to prevent renal fibrosis induced by Ad at 4 weeks.

Although, some studies showed that treatments with TNF-*α* inhibitors have shown protective effects in the models of acute kidney injury (AKI) such as ischemia/reperfusion (I/R) injury [23, 24], but there are few evidences about the effects of TNF-*α* blockers in the models of chronic kidney damage [25, 26]. Recently, a study of an 8-week ETA treatment in mice with aristolochic acid (AA) nephropathy as a model of kidney fibrosis found that ETA partially but significantly attenuated kidney fibrosis and ameliorated albuminuria without affecting kidney function [14]. As previously mentioned, in our study, although we found an improvement in some renal function parameters and observed less tissue damage, we did not find a significant reduction in renal fibrosis with ETA treatment. This could be because the protective effects of TNF-*α* blockers could be more effective in the models of acute damage or using higher doses. Besides that, several factors participate in the pathophysiology of CKD: initiation (proinflammatory cytokines such as TNF-*α*, IL-6, oxidative stress, and TGF-*β*), transition (TGF-*β*, CTGF, and NF-*κ*b), and establishment (TGF-*β*, activation of myofibroblasts, ECM, and collagen types I, II, and IV) where multiple profibrogenic molecules participate [27, 28].

## 5. Conclusion

Treatment with ETA reduces circulating TNF-*α* levels and the severity of adenine-induced tubular damage prior to the establishment of the CKD model. However, inhibition of TNF-*α* is not sufficient to avoid the progression of kidney damage to fibrosis. Actually, it has been widely reported that establishment of fibrosis is a complex phenomenon that ultimately depends on several proinflammatory/anti-inflammatory balance, as well as tissue remodeling molecules (metalloproteinases, integrins, growth factors, etc.), including many other regulators, involving a highly orchestrated event that determines tissue homeostasis, as well as the initiation of inflammation, reinforcement, and perpetuation. In addition, other factors like time of exposition, concentration, and elimination of the nephrotoxic etiological agent compromise the efficiency to carry out the removal of the extracellular matrix. Therefore, although inhibition of TNF by ETA is effective in blocking TNF-*α*, this strategy was partially effective in preventing Ad-induced CKD.

## Figures and Tables

**Figure 1:** Serum TNF-*α* levels. TNF-*α* concentration is shown in the different groups. Ad administration significantly increased serum TNF-*α* levels from the second week, and they remained high until the fourth week of Ad administration compared to the control. Treatment with ETA (Ad+ETA) significantly decreased TNF-*α* concentrations from week 2 to week 4, compared to the Ad groups without treatment. Values are represented as the means ± SEM, *n* = 8. ^∗^*P* < 0.05. Ad: adenine; ETA: etanercept.

**Figure 2:** Kidney morphology and weight gain. (a) Photographs representative of the kidneys at 2 and 4 weeks. Image shows altered color, texture, and a progressive enlargement of the kidneys in groups with Ad. ETA treatment improves the appearance of the kidneys. (b) All animals with Ad administration lose body weight, but animals treated with ETA lose less body weight. (c, d) Kidney reaching a significant enlargement in animals with Ad. ETA treatment reduces the increase in kidney weight and size. Values are represented as the means ± SEM, ^∗^*P* < 0.05. Ad: adenine; ETA: etanercept.

**Figure 3:** Biochemical parameters of kidney function: (a) serum creatinine, (b) serum urea, (c) BUN, (d) urinary creatinine, and (e) urinary volume. Values are represented as the means ± SEM, ^∗^*P* < 0.05. Ad: adenine; ETA: etanercept.

**Figure 4:** Kidney histology. (a) Hematoxylin and eosin stain. Normal kidney architecture was observed in control animals. Interstitial inflammatory infiltrates, crystalline tubulointerstitial deposits, and tubular atrophy are showed in the Ad groups. A partial decrease of interstitial inflammatory infiltrates and tubular atrophy was observed after ETA treatment. (b) Thy-1/DAPI immunostain. The Ad-CKD group exhibited less Thy-1 expression (tubular atrophy), whereas ETA treatment partially maintains the expression of Thy-1 (3 cortical fields per animal were analyzed) (40x). Scale bar is 20 *μ*m. (c) Masson's trichromic staining showed extracellular matrix accumulation in the Ad groups. ETA does not reduce kidney fibrosis at 4 weeks. All are representative photomicrographs of kidney sections in an approximation of 40x.

**Table 1:** Hematological parameters and glomerular filtration rate.

Parameter	Control	Ad	Ad+ETA	Ad	Ad+ETA
		2 w		4 w	
Erythrocytes (10^6^/ml)	7.7 ± 0.1	7.6 ± 0.3	7.60 ± 0.2	6.9 ± 0.0^∗^	6.9 ± 0.1^∗^
Hemoglobin (g/dl)	14.4 ± 0.3	14.1 ± 0.6	14.01 ± 0.4	13.2 ± 0.1^∗^	13.1 ± 0.3^∗^
Hematocrit (%)	42.1 ± 0.9	40.1 ± 1.7	40.2 ± 1.3	38.4 ± 0.3^∗^	38.2 ± 0.8^∗^
Glomerular filtration rate (GFR) (ml/min/g kidney)	0.266 ± 0.03	0.13 ± 0.02^∗^	0.23 ± 0.09	0.02 ± 0.01^∗^	0.04 ± 0.01^∗^

^1^Values are represented as the means ± SEM. ^∗^*P* < 0.05. Ad: adenine; ETA: etanercept.

## Data Availability

All data generated or analyzed during this study are included in this article and/or its supplementary material files. Further inquiries can be directed to the corresponding author.
